# Production, purification and evaluation of biodegradation potential of PHB depolymerase of *Stenotrophomonas* sp. RZS7

This article has been retracted.

**DOI:** 10.1371/journal.pone.0220095

**Published:** 2020-01-07

**Authors:** R. Z. Sayyed, S. J. Wani, Abdullah A. Alarfaj, Asad Syed, Hesham Ali El-Enshasy

**Affiliations:** 1 Department of Microbiology, PSGVP Mandal’s, Arts, Science, and Commerce College, SHAHADA, Maharashtra, India; 2 Department of Botany and Microbiology, College of Science, King Saud University, Riyadh, Saudi Arabia; 3 Institute of Bioproducts Development (IBD), Universiti Teknologi Malaysia (UTM), Johor Bahru, Johor, Malaysia; 4 City of Scientific Research and Technology Applications, New Burg Al Arab, Alexandria, Egypt; North Eastern Regional Institute of Science and Technology, INDIA

## Abstract

There are numerous reports on poly-β-hydroxybutyrate (PHB) depolymerases produced by various microorganisms isolated from various habitats, however, reports on PHB depolymerase production by an isolate from plastic rich sites scares. Although PHB has attracted commercial significance, the inefficient production and recovery methods, inefficient purification of PHB depolymerase and lack of ample knowledge on PHB degradation by PHB depolymerase have hampered its large scale commercialization. Therefore, to ensure the biodegradability of biopolymers, it becomes imperative to study the purification of the biodegrading enzyme system. We report the production, purification, and characterization of extracellular PHB depolymerase from *Stenotrophomonas* sp. RZS7 isolated from a dumping yard rich in plastic waste. The isolate produced extracellular PHB depolymerase in the mineral salt medium (MSM) at 30°C during 4 days of incubation under shaking. The enzyme was purified by three methods namely ammonium salt precipitation, column chromatography, and solvent purification. Among these purification methods, the enzyme was best purified by column chromatography on the Octyl-Sepharose CL-4B column giving optimum yield (0.7993 Umg^-1^mL^-1^). The molecular weight of purified PHB depolymerase was 40 kDa. Studies on the assessment of biodegradation of PHB in liquid culture medium and under natural soil conditions confirmed PHB biodegradation potential of *Stenotrophomonas* sp. RZS7. The results obtained in Fourier-Transform Infrared (FTIR) analysis, High-Performance Liquid Chromatography (HPLC) study and Gas Chromatography Mass-Spectrometry (GC-MS) analysis confirmed the biodegradation of PHB in liquid medium by *Stenotrophomonas* sp. RZS7. Changes in surface morphology of PHB film in soil burial as observed in Field Emission Scanning Electron Microscopy (FESEM) analysis confirmed the biodegradation of PHB under natural soil environment. The isolate was capable of degrading PHB and it resulted in 87.74% biodegradation. A higher rate of degradation under the natural soil condition is the result of the activity of soil microbes that complemented the biodegradation of PHB by *Stenotrophomonas* sp. RZS7.

## Introduction

Poly-β-hydroxy alkanoates (PHAs) or PHB are accumulated as a source of food and energy by a wide variety of bacteria growing under nitrogen stress but carbon-rich conditions isutilized during starvation by the activity of PHB depolymerase [1–3]. PHAs/PHB are considered as the best environment-friendly and renewable option to the synthetics petrochemical plastics because of its similar properties to synthetic plastic [4–6] besides being thermoplastic and biodegradable in nature. Because of such useful properties, it has attracted commercial interest for use as the best alternative to the hazardous synthetic petrochemical polymers and hence it has been successfully commercialized [7–8]. During the last decades much research has been devoted towards the distribution and occurrence of PHB degraders and studies on different PHB depolymerases. Jendrossek and Handrick [9] reported that PHB depolymerases are responsible for extracellular PHB degradation. Extracellular PHB depolymerases of *Aspergillus fumigatus* Pdf1 [10], *Aureobacterium saperdae* [11], *Thermus thermophiles* HB8 [12], *Streptomyces bangladeshensis* 77T-4 [13], *Penicillium simplicissimum* LAR13 [14], *Acidovorax* sp. TP4 [15], *Streptomyces* KJ-72 [16] have been isolated and purified.

There are many different degradation mechanisms that are combined synergistically in nature to degrade polymers [17]. These mechanisms include biodeterioration, biofragmentation, assimilation, mineralization, and enzymatic degradation through extracellular and intracellular depolymerases that break the polymer to water-soluble products. [17]. PHB depolymerases produced by PHA degrading microorganism excrete under starved conditions, which degrade the polymer to water-soluble product forming clearing zones around the PHB depolymerase producing colonies. The action of PHB depolymerase breaks the ester bonds in PHB to produces PHB dimer and 3HB monomer. [18].

The bacterial isolate obtained from the plastic contaminated habitat that possess the ability to degrade PHB may be a potential source of commercially valuable PHB depolymerase, provided that the production, recovery, and purification protocols are properly optimized for large scale production of PHB depolymerase. Therefore, to ensure the biodegradability of biopolymers, it becomes imperative to study the purification of PHB biodegrading enzyme system [16]. PHB depolymerase of isolates obtained from plastic rich habitat is expected to have better relevance for its application in plastic/ bioplastic degradation.

The present paper reports the production, purification, and characterization of extracellular PHB depolymerase of *Stenotrophomonas* sp. RZS7 isolated from a plastic contaminated site in North Maharashtra region of India.

## Materials and methods

### PHB

PHB procured from Sigma-Aldrich, Germany was used as a standard for all experiments.

### Source of cultures

Cultures of fungi; *Aspergillus niger* NCIM1025, *A*. *flavus* NCIM650, *Alternaria alternate* ARI715, and *Cercospora arachichola* were procured from NCIM, NCL, Pune, Maharashtra, India. *Alcaligenes* sp RZS4 and *Pseudomonas* sp. RZS1 and *Streptomycetes* sp. were obtained from the culture depository of the Department. For present study, *Stenotrophomonas* sp. RZS7 that was previously identified [19] was used as PHB depolymerase producer.

### Production of PHB depolymerase

Production of PHB depolymerase was carried out by shake flask method by growing *Stenotrophomonas* sp. RZS7 in MSM containing (gL^-1^) PHB, 0.015 K_2_HPO_4_, 0.07 g; KH_2_PO_4_, 0.07 g; MgSO_4_, 0.07 g; NH_4_Cl, 0.1 g; NaNO_3_, 0.1 g; NaCl, 0.5 mg; FeSO_4_, 0.2 mg, ZnSO_4_, 0.7 mg [14] at 120 rpm for 4 days at 30°C.

### PHB depolymerase assay

Following the incubation, MSM was centrifuged a 10,000 rpm for 15 min and the supernatant was used for PHB depolymerase assay [12]. The reaction mixture contained 150 μg ml^-1^ PHB granules, (substrate for PHB depolymerase) and 2 mM CaCl_2_ 50 mM Tris-HCl buffer (pH 7.0) and 0.5 mL of supernatant from MSM. Enzyme activity was spectrophotometrically measured at 650 nm as a decrease in the PHB turbidity. One unit of PHB depolymerase was defined as the quantity of enzyme required to decrease the absorbance by 0.1 min^-1^.

### Purification of PHB depolymerase

The cell-free supernatant of, MSM was subjected for purification of the enzyme as follows -

#### Ammonium salt precipitation

The cell-free supernatant was precipitated by adding increasing concentration (10–80% w/v) of solid ammonium sulfate with continuous stirring at 4°C for 1 h. The precipitate was dissolved in the Tris-HCl buffer (pH 7), supernatant and the dissolved precipitate was transferred in a separate dialysis bag and allowed for overnight dialysis in chilled phosphate buffer (pH 7.0) [13]. The protein content of dialyzed supernatant and dialyzed precipitate was measured as per Lowry et. al. method [20]. PHB depolymerase activity of dialyzed supernatant and dialyzed precipitate was measured [12].

#### Solvent purification method

The cell free supernatant was centrifuged at 10,000 rpm for 20 min. The residue obtained was dissolved in pre-chilled 1:1 acetone ethanol mixture, shaken well and kept in a water bath at 50°C until all solvent is evaporated. The pellet obtained after evaporation was dissolved in Tris-HCl buffer (pH 7). PHB depolymerase activity of pellet and supernatant was measured [12].

#### Column chromatography

The cell-free supernatant obtained from MSM was loaded onto an Octyl-Sepharose CL-4B column pre-equilibrated with 50 mM glycine NaOH buffer (pH 9.0) followed by elution with 50% ethanol [12]. The eluting fractions were separately collected and subjected for PHB depolymerase [12].

### Determination of molecular weight of purified PHB depolymerase

Determination of the molecular weight of purified PHB depolymerase was performed by Sodium Dodecyl Sulfate Polyacrylamide Gel Electrophoresis (SDS-PAGE). Purified fractions and standard protein marker (Ge-Nei, Bangaluru, India) were electrophoresed at 50 mv for 2 h. The separated bands were stained with Coomassie Brilliant Blue R-250 and visualized under UV transilluminator. The separated bands of test protein were compared with standard protein markers. The proteins content of bands was estimated by as per Lowry et al. [20].

### Assessment of biodegradation of PHB

To evaluate the efficacy of degradation of biopolymer, the following methods were used

#### PHB biodegradation under laboratory conditions

Preparation of PHB film was done as per Linag et al. [21].PHB powder (0.15 gm) was dissolved in 50 mL chloroform and vortexed for 10–15 min. The solution was poured into clean, dry Petri dishes and kept overnight at30°C. PHB film was obtained following the evaporation of chloroform. This film was used for the assessment of biodegradation.

PHB film was separately added as a sole carbon source into MSM and inoculated with *Stenotrophomonas* sp. RZS7 and incubated at 30°C for 10 days at 120 rpm and observed for degradation of PHB film. Qualitative estimation involved the weight loss method. Quantitative estimation involved the measurement of change in optical density and crotonic acid concentration (μgmL^-1^) at a different time intervals at 235 nm, [22]. The amount of crotonic acid was calculated from the calibration curve prepared with standard crotonic acid in the range of 10–100 μgmL^-1^.

#### PHB biodegradation under natural soil conditions

Soil burial test gives an indication of the biodegradation of the polymer in a given soil under specific conditions. To check the biodegradability and durability of polymer sample under natural soil conditions, soil burial test was carried out. For this purpose garden soil was taken in different trays (1800 gm per tray) and the PHB film covered with the net was incorporated into the tray with *Stenotrophomonas* sp. RZS7 and trays were covered with moist thick paper [23]. Degradation of PHB film by *Stenotrophomonas* sp. RZS7 was observed in five different sets and was compared with negative control containing only sterile soil. The degradation of PHB film was measured in terms of weight loss and was expressed as percent reduction in the weight of PHB film

### Fourier-transform infra red (FTIR) spectroscopy analysis

Following the desired incubation period for degradation, the inoculated and incubated liquid culture medium of *Stenotrophomonas* sp. RZS7 was subjected to FTIR analysis on FTIR (FTIR Model 8400S, Shimadzu, Japan,) by using IR solution version 1.40 software. FTIR spectra were read between 4000 to 500 cm^-1^ [24]. The functional groups present in degradation patterns were determined by FTIR and compared with the control.

### High-performance liquid chromatography (HPLC) analysis

HPLC analysis of the preparation was analyzed on HPLC (Younglin, South Koria, ACME-9000) [25]. For this purpose, 20 μL of sample was injected into the C18 column as stationary phase and allowed to run 0.6 mL min^-1^ on a mobile phase of acetonitrile: water (30:70 v/v) at 254 nm. The peaks were analyzed by using Autochro-3000 software.

### Gas chromatography-mass spectroscopic (GC-MS) analysis

#### Sample preparation

The cell-free supernatant (2 mL) from a liquid medium was mixed with 2 mL chloroform and 2 mL of acidified methanol. For depolymerization and methanolysis of PHB, the mixture was heated at 100°C for 3 h with occasional shaking followed by subsequently cooling at 30°C followed by heating at 100°C for 3 h and adding 1 mL of distilled water. The whole content was vortexed for 2 min and allowed to stand for 10 min to separate the phases. At the bottom layer, organic phase was obtained by a glass Pasteur pipette and it was subjected for spectral analysis [26].

#### GC-MS analysis

Monomers present in the degraded sample were identified by GC-MS (Model Autosystem XL, Perkin Elmer, USA) equipped with an SGE forte GC capillary column BP20 (Australia) and mass spectrophotometer. The mass spectra obtained were compared with the spectra of standard methyl esters of PHB available from mass spectra library of the National Institute of Standards and Technology (NIST), USA. The peak identities were initially identified based on their matching of relative retention time with respect to standard sample extracted at time zero.

#### GC-MS parameters

One μL of sample was injected with a split ratio of 10:1. The rate of flow of carrier gas (helium) was 1 mL min^-1^. The oven temperature of the column was programmed from 120°C for 2 min, increased at a rate of 20°C min^-1^ to 230°C, and held at this temperature for 10 min. The temperature of the injector and detector was 225°C and 230°C respectively.

### Field emission scanning electron microscopy (FE SEM) analysis

FE SEM was used to study the surface morphology and structural changes in PHB film following the biodegradation in soil burial test. PHB film from soil burial sample was thoroughly washed with sterile distilled water and mounted on stub using carbon tape it was made conducting by gold coating in vacuum by evaporation. The polymer film was dried in an Infrared (IR) lamp. The images of the treated test samples and untreated test samples were compared.

### Statistical analysis

Three replicates of each experiment were run and the average value of triplicates was recorded. The data was analyzed by Student’s *t-*test and values of *P* ≤ 0.05 were taken as statistically significant [27].

## Results and discussion

### Production of PHB depolymerase

After 4 days of incubation at 30°C at 120 rpm in MSM, *Stenotrophomonas* sp. RZS7 yielded 0.721 U mL^-1^ PHB depolymerase. Similar enzyme activities have been reported by other researchers [21,28]

### Purification of PHB depolymerase

#### Ammonium salt precipitation

Protein precipitation was increasing with increase in the concentrations of ammonium sulfate in the cell-free supernatant of *Stenotrophomonas* sp. RZS7, maximum proteins were precipitated with 70% ammonium sulfate concentration (Table 1). The protein concentration, specific activity and enzyme activity of PHB depolymerase in the dialyzed precipitate of *Stenotrophomonas* sp. RZS7 were 0.219 mgmL^-1^, 0.7031 Umg^-1^mL^-1^ and 0.154 UmL^-1^ respectively. Zhou et al. [28] have precipitated PHB depolymerase of *Escherichia coli*, and *Penicillium* sp. DS9701-D2 in 70 and 75% of ammonium sulfate respectively. Shivkumar et al. [29] have purified PHB depolymerase of *Penicillium citrinum* S2 in 80% of ammonium sulfate.

**Table 1:** Purification profile of PHB depolymerase by various methods.

Purification method	Enzyme activity (Umg-^1^mL^-1^)
Salt precipitation	0.7031 (0.090)
Solvent purification	0.1120 (0.022)
Column chromatography	0.7993 (0.099)

Values are statistically significant at P ≤ 0.05

Values are the mean of triplicates

Values in the parenthesis are standard deviation

#### Solvent purification method

Solvent purification of PHB depolymerase of *Stenotrophomonas* sp. RZS7 retained only 51.14% and 38.81% enzyme activity in pellet and supernatant (Table 1).

The protein concentration, specific activity and enzyme activity of PHB depolymerase in pellet and supernatant were 0.219 mgmL^-1^, 0.5114 Umg^-1^mL^-1^, and 0.3881 UmL^-1^ respectively. The loss of enzyme activity in solvent system is due to the denaturation of proteins caused by the solvent system. Thus the solvent purification method proved an ineffective for purification of PHB depolymerase of *Stenotrophomonas* sp. RZS7.

#### Column chromatography

A total of five fractions were obtained from Octyl-Sepharose CL-4B. Among all the fractions analyzed for PHB depolymerase enzyme activity, the 3^rd^ fraction showed maximum enzyme activity (Table 2). PHBV depolymerase of *Bacillus* sp. AF3 and *Streptoverticillium kashmirense* AF1 have also been purified on Sephadex G-75 [30]. Kim et al. [31] have also purified PHB depolymerase of *Emericellopsis minima* W2 and *Streptomyces* sp. KJ-72 on Sephadex G-100 and Sephadex G-150 respectively. Papaneophytou et al. [12] and Hsu et al. [13] have isolated and purified extracellular PHB depolymerases of *Thermus thermophiles* HB8 and *Streptomyces bangladeshensis* 77T-4 respectively using column chromatography.

**Table 2:** Purification of PHB depolymerase of *Stenotrophomonas* sp. RZS7 on Octyl sepharose column.

Fraction	Total activity (UmL^-1^)	Total protein (mgmL^-1^)	Specific activity (U mg^-1^mL^-1^)	% activity
1	0.027 (0.027)	0.031 (0.010)	0.0782 (0.032)	11.13 (0.012)
2	0.101 (0.011)	0.153 (0.037)	0.3781 (0.041)	48.31 (0.039)
3	0.247 (0.015)	0.309 (0.074)	0.7993 (0.090)	79.93 (0.092)
4	0.017 (0.001)	0.015 (0.009)	0.0106 (0.011)	04.01 (0.012)
5	0.003 (0.001)	0.006 (0.005)	0.0011 (0.008)	00.10 (0.002)

Values were statistically significant at P ≤ 0.05

Values in the parenthesis are standard deviation

Among all three purification methods, purification on Octyl sepharose CL-4B column gave good purification yield (Table 1), more enzyme activity and more specific activity. The protein concentration, specific activity and enzyme activity of PHB depolymerase were 0.309 UmL^-1^, 0.7993 Umg-1 mL-1 and 0.247 mgmL-1 respectively.

### Determination of molecular weight of purified PHB depolymerase

The protein fraction of *Stenotrophomonas* sp. RZS7 obtained from the octyl sepharose CL-4B column that exhibited maximum enzyme activity revealed a single protein band in SDS PAGE having a molecular mass of about 40 kDa Sadocco et al. [11] have also reported the molecular mass of 42.7 kDa PHB depolymerase in *Aureobacterium saperdae*.

### Assessment of biodegradation of PHB

Among the various reference cultures taken from our own departmental culture depository; all fungal and bacterial cultures were unable to degrade PHB when growing in PHB containing MSM. However, only *Streptomycetes* sp. was found to degrade PHB on 10^th^ day of incubation but the extent of PHB biodegradation in this case was less. Hence for further biodegradation studies *Stenotrophomonas* sp. RZS7 was used.

#### Qualitative measurement

A gradual reduction in the weight of PHB film was recorded after 8 days of incubation fragmentation in PHB film was observed while no changes occurred in a control sample of PHB film (Table 3). Varda et al. [32] have recorded similar loss of weight of starch-based plastic by *S*. *epidermidis*.

**Table 3:** Qualitative measurement of biodegradation of PHB film.

Weight of PHB film	Weight loss of PHB film (g)	OD	Crotonic acid* (μgmL^-1^)
Initial weight	0.159 (0.031)	0.000	1000 0.030)
After 2 days	0.148 (0.029)	0.014	813 (0.026)
After 4 days	0.109 (0.021)	0.019	794 (0.019)
After 6 days	0.099 (0.017)	0.035	705 (0.018)
After 8 days	Fragmentation	0.050	686 (0.015)

Values were statistically significant at P ≤ 0.05

Values in the parenthesis are standard deviation

*Crotonic acid was as PHB standard for spectrophotometric estimation of PHB as when PHB is heated with concentrated sulphuric acid it gets converted into crotonic acid.

#### Quantitative estimation

Isolate RZS7 caused the reduction in the amount of crotonic acid with an increase in the biomass. The maximum reduction in the amount of crotonic acid was recorded on 10^th^ day of incubation at 37°C (Table 3). The reduction in crotonic acid concentration can be taken as the evidence of biodegradation of PHB film.

### Fourier transform infrared (FTIR) spectroscopy analysis

FTIR analysis of liquid culture medium containing PHB film and inoculated with *Stenotrophomonas* sp. RZS7 showed changes in the functional groups and significant shift of wavenumbers, indicating the biodegradation of polymer. It was observed that in case of control preparation (without inoculum) FTIR chromatogram peaks appearing at 3020.63 cm^-1^ changed to 3018.70, 2926.11, 2856.67 cm^-1^, 2399.53 cm^-1^ changed to 2360.95, 2333.94 cm^-1^, 2088.98 cm^-1^ changed to 2079.33 cm^-1^, 1641.48 cm^-1^ shifted to 1629.90 cm^-1^ and 1631.83 cm^-1^ shifted towards 1529.60, 1427.37, 1381.08 cm^-1^ (Figs 1 and 2). The major functional groups in control sample were found at wavelength frequency 1641.48 and 1631.83 denoted C = O stretch in ketone, frequency 3020.63 denoted C-H which stretch in alkane, wavelength frequency 1014.59 denoted C-O which stretch in ester and 756.12 denoted C-H which is rock alkane. However the major functional group frequency changes observed in degrading sample i.e. 1629.90 denoted C = O which stretch in ketone, 1215.19 which denote alkyl halide, 2399.53,2360.95 and 2333.94 denoted H-C = O group, 927.79 denoted C-O which stretch in ester, 769.62 denoted C-H which is rock alkane. These changes in wavelength frequency of major functional groups in degrading samples as compared to control give preliminary proof of biodegradation of polymer by *Stenotrophomonas* sp. RZS7.

**Fig 1:** **FTIR chromatogram of PHB (Control)** read between 4000 to 500 cm^-1^ and analyzed with 1.40 software.

**Fig 2:** **FTIR chromatogram of PHB after degradation by *Stenotrophomonas* sp.** RZS7 read between 4000 to 500 cm^-1^ and analyzed with 1.40 software. The functional groups present in the spectra were compared with the functional groups in control preparation.

### High performance liquid chromatography (HPLC) analysis

The spectra of the original polymer sample before degradation revealed six peaks at 254 nm (Fig 3). While polymer sample degradation by *Stenotrophomonas* sp. RZS7 revealed nine peaks having different retention time as compared to control (Fig 4) indicating the formation of monomers. The sum of the total area of peaks of the degraded sample was less than the sum of the total area of peaks of control (undegraded) preparation. This reduction in the peak area confirmed the degradation of the polymer.

**Fig 3:** HPLC spectra of polymer before degradation (Control) recorded at 254 nm). Spectral analysis was carried out at 254 nm with autochro-3000 software.

**Fig 4:** HPLC spectra of polymer after degradation recorded at 254 nm. The peaks were analyzed by using Autochro-3000 software and compared with the peaks of control.

### Gas chromatography-mass spectroscopic (GC-MS) analysis

The degradation pattern on the basis of removal or decrease in the retention time of the peaks and their comparison with the retention time of the peaks of reference demonstrated the disappearance of peaks indicating biodegradation of PHB components by *Stenotrophomonas* sp. RZS7 (Fig 5 and Fig 6). A significant decrease in area height and percentage in the degraded sample was clear over the control (undegraded) sample. The total area of peaks of degraded sample was less as compared to the total area of peaks of control (undegraded) preparation. This reduction in the peak area confirmed the conversion of PHB due to its biodegradation into monomers.

**Fig 5:** Chromatogram of polymer sample before biodegradation (Standard). GC MS analysis was performed on gas chromatograph equipped with capillary column BP20 and mass spectrophotometer. The mass spectra obtained were recorded.

**Fig 6:** Chromatogram of polymer sample after biodegradation. GC MS analysis was performed by using gas chromatograph with turbomass GC capillary column BP20 and mass spectrophotometer. The mass spectra obtained were compared and identified with the library of spectra of standard methyl esters of PHB. The peaks were identified by matching relative retention time with respect to standard sample extracted at time zero.

The fragmentation patterns with GC-MS and the identities of peaks in the mass spectra were correlated to the carbonyl and hydroxyl ends of the represented hydroxyl alkanoates ethyl esters of PHB after degradation. Tridecanoic acid 12-methyl-methyl ester and heptacosanoic acid methyl ester in standard polymer sample were completely degraded whereas Decanoic acid methyl ester, undecanoic acid methyl ester, and nonanoic acid methyl ester were detected in the degraded sample (Table 4). McLafferty and Turecek [33] reported that the mass spectra of the methyl esters of PHB dominated by m/z = 74 represented the carbonyl end of the molecule and showed the characteristic of 3-hydroxyl functional groups. However, the peak at m/z = 59 indicated the release of the hydroxyl end during the cleavage of the molecule between C3 and C4.

**Table 4:** GC MS analysis of methanolysed polymer before degradation (Standard) and after degradation.

Retention time	Methyl ester PHB monomers (before degradation)	MW	Methyl ester PHB monomers (after degradation)	MW
	Pentadecanoic acid, 14-methyl-, methyl ester Hexadecanoic acid, methyl ester	270	Tridecanoic acid, methyl ester	228
	Tridecanoic acid, methyl ester	228	Pentadecanoic acid, 14-methyl-, methyl ester Hexadecanoic acid, methyl ester	270
	Hexadecanoic acid, 15-methyl-, methyl ester Heptadecanoic acid, methyl ester	284	Hexadecanoic acid, 15-methyl-, methyl ester Heptadecanoic acid, methyl ester	284
	Heneicosanoic acid, methyl ester	340	Decanoic acid, methyl ester	186
	Docosanoic acid, methyl ester	354	Dodecanoic acid, methyl ester	214
	Eicosanoic acid, methyl ester	326	Undecanoic acid, methyl ester	200
	Hexacosanoic acid, methyl ester	410	Methyl tetradecanoate	242
	Methyl tetradecanoate Tridecanoic acid, 12-methyl-, methyl ester	242	Pentadecanoic acid, methyl ester	256
	Octadecanoic acid, methyl ester	298	Eicosanoic acid, methyl ester	326
	Dodecanoic acid, methyl ester	214	Heneicosanoic acid, methyl ester	340
	Pentadecanoic acid, methyl ester	256	Octadecanoic acid, methyl ester	298
	Heptacosanoic acid, methyl ester	424	Docosanoic acid, methyl ester	354
			Hexacosanoic acid, methyl ester	410
			Nonanoic acid, methyl ester	172

The mass spectra of standard polymer sample and the characteristics signals were recorded at m/z = 29, 39, 41, 43, 45, 55, 57, 59, 74, 75, 87, 101, 111, 131, 143, 157, 171, 185, 199, 219, 227, 239, 265, 270, 271, 314, 415. However in polymer degrading sample m/z = 29, 32, 41, 43, 44, 55, 57, 69, 74, 75, 87, 97, 111, 129, 143, 145, 169, 176, 199, 220, 227, 270 (Fig 7) which can be attributed to oligomers of PHB (Fig 8). Wennan et al. [34] reported that m/z = 29, 32, 41, 43, 55, 69, 75, 87, 97, 111, 143 denotes Pentadecanoic acid methyl ester, m/z = 29, 41, 55, 57, 69, 74, 75, 87, 97 denotes Decanoic acid, methyl ester, m/z = 41, 43, 55, 74 denotes Dodecanoic acid methyl ester, m/z = 74 denotes Hexadecanoic acid methyl ester, m/z = 43, 55, 74 denotes Octadecanoic acid methyl ester.

**Fig 7:** GC-MS spectra of polymer sample before degradation showing mass spectra of m/z = 29, 39, 41, 43, 45, 55, 57, 59, 74, 75, 87, 101, 111, 131, 143, 157, 171, 185, 199, 219, 227, 239, 265, 270, 271, 314, 415 indicating the presence of intact polymer of PHB.

**Fig 8:** GC-MS spectra of polymer sample after degradation showing mass spectra of m/z 29, 32, 41, 43, 44, 55, 57, 69, 74, 75, 87, 97, 111, 129, 143, 145, 169, 176, 199, 220, 227, 270 indicating the presence of oligomers of PHB.

### Field emission scanning electron microscopy (FE-SEM) analysis

Surface analysis of PHB film after soil burial experiment showed many differences in the morphology of PHB film as compared to control (Fig 9A) and PHB film buried in the soil (Fig 9B). Biodegradation of PHB film caused erosion and roughening of the surface of PHB film (Fig 9C). Gautam and Kaur [35] have also reported the morphological changes in polyethylene surface after degradation as compared with control. Calabia and Tokiwa [36] analyzed the degradation of PHB by SEM and observed the presence of holes on the surface of PHB film due to the growth of *Streptomyces* sp. SC-17 on the surface of PHB film causing biodegradation of PH B.

**Fig 9:** Morphological changes in PHB film after soil burial test observed under FE SEM; (A) Control set, (B) PHB film buried in presence of natural soil, (C) PHB film degraded by *Stenotrophomonas* sp. RZS7.

## Conclusion

The present attempt provided PHB degrading *Stenotrophomonas* sp. RZS 7 which utilized PHB as a sole source of carbon under the influence of extracellular PHB depolymerase. The enzyme acted as a key enzyme responsible for the biodegradation of PHB. Purification of PHB depolymerase by solvent purification resulted in protein precipitation and denaturation of the enzyme. Column chromatography appeared as an efficient and best purification method as it yielded maximum protein, maximum enzyme activity, and maximum specific activity. The molecular weight of purified PHB depolymerase of *Stenotrophomonas* sp. RZS7 (40 kDa) matched with a molecular weight of *Aureobacterium saperdae*.

Biodegradation of PHB in liquid culture medium and under natural soil conditions confirmed PHB biodegradation potential of *Stenotrophomonas* sp. RZS7. The results obtained in FTIR analysis, HPLC study and GC-MS analysis confirmed the biodegradation ability of *Stenotrophomonas* sp. RZS7 in liquid medium. Changes in surface morphology of PHB film in the soil burial as observed in FE SEM analysis confirmed the ability of isolate to degrade PHB under natural soil conditions. Higher rate of degradation under natural soil condition is the result of activity of soil microbes that complemented the degradation by *Stenotrophomonas* sp. RZS7.
